The article "Colonic Angiolipoma: An Extremely Rare Tumor Clinically Masquerading as Acute Appendicitis" was retracted in 2024. Reasons: false authorship; unreliable results or conclusions; no approval from an author; concerns about the authorship.

# Colonic Angiolipoma: An Extremely Rare Tumor Clinically Masquerading as Acute Appendicitis

**DOI:** 10.7759/cureus.20659

**Published:** 2021-12-24

**Authors:** Abdullah S Alfaraj, Asma A Almohamad, Nader S Alqabbani, Mohammed H Alghazwi, Abdulkarim M Alharbi, Amina A Ahmed, Marwan K Aljumah, Naif Y Aljumaah, Hawra E Kadhem, Hassan H Al Jalooud, Zahra S AlMohsen, Kawkab M Alharbi, Hassan E Al Abbas, Fatimah B Al Khalifah, Faisal Al-Hawaj

**Affiliations:** 1 General Practice, Al Naeriyah Hospital, Naeriyah, SAU; 2 College of Medicine, Ibn Sina National College for Medical Studies, Jeddah, SAU; 3 College of Medicine, Arabian Gulf University, Manama, BHR; 4 College of Medicine, Prince Sattam Bin Abdulaziz University, Al-Kharj, SAU; 5 College of Medicine, King Saud University, Riyadh, SAU; 6 College of Medicine, Xi'an Jiaotong University, Xi'an, CHN; 7 College of Medicine, Qassim University, Qassim, SAU; 8 College of Medicine, Vision College, Riyadh, SAU; 9 College of Medicine, King Faisal University, Hofuf, SAU; 10 College of Medicine, Princess Nourah Bint Abdulrahman University, Riyadh, SAU; 11 College of Medicine, Imam Abdulrahman Bin Faisal University, Dammam, SAU

**Keywords:** case report, abdominal pain, laparoscopy, lipoma, angiolipoma, acute appendicitis

## Abstract

The clinical presentation of right iliac fossa pain, anorexia, and vomiting are the classic clinical features of acute appendicitis. However, a broad spectrum of manifestations may result in a similar clinical picture, including gastrointestinal, genitourinary, and gynecologic pathologies. Imaging studies are crucial to establishing the diagnosis. Here, we report the case of a 58-year-old man who presented to the emergency department with a one-week history of right lower quadrant abdominal pain. The pain was associated with nausea, vomiting, and frequent bowel motions. There was no history of fever or weight loss. The examination of the abdomen showed localized tenderness and guarding in the right iliac fossa. The basic laboratory investigation was within the reference range. The computed tomography scan demonstrated a well-circumscribed intraluminal mass lesion in the ascending colon with no evidence of complete obstruction. The mass was slightly heterogeneous but had fat attenuation. There was no evidence of invasion. There was no stranding of the adjacent fat. The radiological findings were consistent with colonic lipoma. The patient underwent laparoscopic surgery and had a segmental resection of the tumor with primary anastomosis. The appendix was also resected. Histopathological examination showed mature adipose cells along with thin-walled, capillary-sized vessels representing a benign angiolipoma. Further, the resected appendix was completely normal and showed no evidence of acute inflammation. Colonic angiolipoma is an extremely rare tumor. This case demonstrated that a large angiolipoma of the ascending colon may show a presenting clinical picture similar to that of acute appendicitis. Complete resection of the tumor is associated with an excellent outcome.

The article "Colonic Angiolipoma: An Extremely Rare Tumor Clinically Masquerading as Acute Appendicitis" was retracted in 2024. Reasons: false authorship; unreliable results or conclusions; no approval from an author; concerns about the authorship.

## Introduction

Acute appendicitis is one the most frequent causes of acute abdomen and is considered one of the major indications for emergency abdominal surgeries worldwide. The classic clinical features of acute appendicitis include right lower quadrant abdominal pain, anorexia, and nausea and vomiting [1]. However, there are several conditions that can mimic acute appendicitis, including a wide range of gastrointestinal, genitourinary, and gynecologic conditions [2]. Hence, imaging with ultrasound or cross-sectional imaging modalities is crucial to confirm the diagnosis and identify possible complications. The gastrointestinal pathologies that may have a similar clinical picture to acute appendicitis include Crohn’s disease, infectious enterocolitis, mesenteric adenitis, acute diverticulitis, Meckel diverticulitis, and epiploic appendagitis [3]. Here, we present the case of a middle-aged patient with classic clinical presentation of acute appendicitis who was diagnosed with colonic angiolipoma, an extremely rare benign tumor of the gastrointestinal tract.

## Case presentation

A 58-year-old man presented to the emergency department with a one-week history of right lower quadrant abdominal pain. He reported that the pain had started in the periumbilical area and shifted to the current location. It had a gradual onset and had been increasing in severity. The pain was sharp in nature and was not related to food intake or posture. He attempted over-the-counter analgesic and antacid medications with no significant clinical improvement. He scored the pain as 7 out of 10 in severity and reported that had it started to disrupt his sleep. The pain was associated with nausea, vomiting, and frequent bowel motions. There was no history of fever or weight loss.

The patient had a longstanding history of metabolic syndrome with hypertension, diabetes mellitus, and dyslipidemia. He had stable angina that was well-controlled with medications. He was diagnosed as having gastroesophageal reflux disease seven years ago. His medications included metformin 500 mg, captopril 25 mg, metoprolol 25 mg, atorvastatin 20 mg, and omeprazole 40 mg. He reported good compliance with his medications, and his allergy history was unremarkable. He had not undergone any surgeries. He worked as a taxi driver and had a smoking history of 18 packs a year. He consumed alcohol on a few occasions only. His family history was remarkable for colon cancer.

The article "Colonic Angiolipoma: An Extremely Rare Tumor Clinically Masquerading as Acute Appendicitis" was retracted in 2024. Reasons: false authorship; unreliable results or conclusions; no approval from an author; concerns about the authorship.

Upon examination, the patient appeared in discomfort. His vital signs were within the normal limits with a heart rate of 88 beats per minute, a temperature of 37.0°C, a respiratory rate of 12 breaths per minute, and blood pressure of 122/84 mmHg. The examination of the abdomen showed localized tenderness and guarding in the right iliac fossa. However, there were no signs of generalized peritonitis. Bowel sounds were present with normal intensity. Digital rectal examination was normal. Other systems showed normal examination findings.

The basic laboratory investigation was within the reference range. In particular, leukocytes, erythrocyte sedimentation rate, and C-reactive protein levels were normal. The liver enzymes, electrolytes, and blood urea nitrogen were also normal (Table 1). The initial diagnosis was acute appendicitis. The patient underwent abdominal computed tomography (CT) to rule out any complication of acute appendicitis as his pain had persisted for one week. The scan demonstrated a well-circumscribed intraluminal mass lesion in the ascending colon with no evidence of complete obstruction. The mass was slightly heterogeneous but had fat attenuation. There was no evidence of invasion. There was no stranding of the adjacent fat. The radiological findings were consistent with a colonic lipoma (Figure 1).

**Table 1:** Summary of the laboratory findings.

Laboratory investigation	Finding
Hemoglobin	14.9 g/dL
White blood cells	8,400/mL
Platelets	386,000/mL
Erythrocyte sedimentation rate	6 mm/hour
C-reactive protein	6.3 mg/dL
Total bilirubin	0.8 mg/dL
Albumin	4.5 g/dL
Alkaline phosphatase	44 U/L
Gamma-glutamyltransferase	23 U/L
Alanine transferase	18 U/L
Aspartate transferase	23 U/L
Blood urea nitrogen	8 mg/dL
Creatinine	0.7 mg/dL
Sodium	136 mEq/L
Potassium	4.1 mEq/L
Chloride	98 mEq/L

**Figure 1:** Axial (A) and coronal (B) CT images showing a slightly heterogeneous fat-density mass lesion (arrow) in the ascending colon. CT: computed tomography

The patient underwent laparoscopic surgery for further evaluation and management. During exploration, the previously seen mass lesion was identified. The appendix had a normal appearance with no congestion to suggest acute appendicitis. Segmental resection of the tumor was performed with primary anastomosis. The appendix was also resected. The recovery of the patient was uneventful. Postoperatively, he reported improvement in his pain. He started oral feeding on the second postoperative day and was tolerating it well. He was discharged on the sixth postoperative day. Histopathological examination showed mature adipose cells along with thin-walled, capillary-sized vessels representing a benign angiolipoma (Figure 2). Further, the resected appendix was completely normal and showed no evidence of acute inflammation. No complaints were reported by the patent during the follow-up visit after three months.

The article "Colonic Angiolipoma: An Extremely Rare Tumor Clinically Masquerading as Acute Appendicitis" was retracted in 2024. Reasons: false authorship; unreliable results or conclusions; no approval from an author; concerns about the authorship.

**Figure 2:** Histopathological examination showing mature adipocytes and blood vessels in keeping with angiolipoma.

## Discussion

We reported the case of a colonic angiolipoma that had a classic presentation of acute appendicitis. Angiolipoma is a rare benign tumor of mature adipose tissue and blood vessels. It typically occurs in the subcutaneous tissue in the trunk and upper extremities in young adults and presents as a tender small nodule. However, colonic angiolipoma is an extremely rare entity with few reported cases in the literature [4-10]. This tumor was first described by Bowen in 1912 [10]. The tumor is classified into lipomatous and angiomatous types according to the predominant histologic component [5]. In the present case, the ratio of vascular tissue and adipose tissue was almost similar.

A recent review of the literature by Kimura et al. [4] in 2021 showed only 15 cases of colonic angiolipoma reported in the English medical literature. Among these, only three cases of angiolipoma occurred in the ascending colon, as in our case. The clinical manifestation of colonic angiolipoma was non-specific. However, the presentation with intussusception was reported in multiple cases [4,5,8]. In our case, the patient presented with the classic clinical presentation of acute appendicitis. We postulate that the location of the tumor in the ascending colon leads to increased luminal pressure proximally resulting in the classic pain of appendicitis. However, the histopathological examination of the appendix was completely normal.

The diagnosis of angiolipoma cannot be made confidently by imaging studies. In our case, the radiological diagnosis was a lipoma. However, it has been reported that on magnetic resonance imaging the tumor shows the signal intensity of adipose tissue along with low T1 signal intensity and high T2 signal intensity in the vascular element that exhibits vivid contrast enhancement [4]. The accurate diagnosis is often confirmed by histopathological examination of the resected specimen [5,8].

Regarding the management of colonic angiolipoma, the method of surgical resection largely depends on the location of the tumor, its type, and size. Endoscopic resection can be performed for small-sized pedunculated tumors [9]. However, partial resection of the tumor is the method of choice in most cases [7]. The tumor is benign and has an excellent prognosis. However, recurrence may occur if it was not resected completely [5]. In our case, examination of the resected specimen showed complete resection, and the patient did not develop any further complaints on the follow-up to suggest recurrence. The laparoscopic approach can be performed for such tumors, as in our case [4].

The article "Colonic Angiolipoma: An Extremely Rare Tumor Clinically Masquerading as Acute Appendicitis" was retracted in 2024. Reasons: false authorship; unreliable results or conclusions; no approval from an author; concerns about the authorship.

## Conclusions

Colonic angiolipoma is an extremely rare tumor. Our case demonstrated that a large angiolipoma of the ascending colon may show a presenting clinical picture similar to that of acute appendicitis. A CT scan may suggest the benign lipomatous nature of the lesion, but the accurate diagnosis of angiolipoma is often made by histopathology. Complete resection of the tumor is associated with an excellent prognosis which can be achieved by laparoscopic procedures.
